# Application of Convolutional Neural Network to GIS and Physics

**DOI:** 10.1155/2022/8559343

**Published:** 2022-07-19

**Authors:** Jinglei Liu, Fangfang Dong, Zhiyao Li

**Affiliations:** ^1^Changwang College, Nanjing University of Information Science and Technology, Nanjing, Jiangsu 210044, China; ^2^Physical Group, Yancheng Tinghu Senior High School, Yancheng, Jiangsu 224051, China; ^3^School of Electronic Engineering, Nanjing Xiaozhuang University, Nanjing, Jiangsu 211171, China

## Abstract

Human life and property are often seriously threatened and lost due to natural disasters such as earthquakes. As a spatial information system, the geographic information system (GIS) can collect, store, and manage the local or whole related physical data of the surface space to be measured with the support of software and hardware. The physical data is collected through GIS for performance testing. The data are collected from the aftershock event records of the Wenchuan earthquake. Among them, 14,000 Wenchuan earthquake events are used as the original data set, and 8,800 aftershock events are used as the test data set. Seismic data involves the detection of multiple physical quantities, which makes the seismic data gradually increase, many data have no obvious linear relationship, and traditional detection methods are difficult to meet the detection requirements. The artificial intelligence method led by a convolutional neural network (CNN) can perform pattern matching on complex nonlinear variables, and models with general characteristics can be generated from different seismic waveforms for the prediction of seismic waveforms. The results show that GIS can effectively intercept and collect seismic physical signals. The training and detection accuracy of CNN combined with GIS physical data is higher than 90%. Compared with traditional training methods, CNN is obviously superior in detection accuracy and recall rate. At the same time, a large number of microseismic events that are easily missed by manual selection can also be found.

## 1. Introduction

Since the 1990s, geographic information system (GIS) technology has been widely used in the domestic earthquake field, and its application fields include earthquake analysis, earthquake resistance, prediction, disaster prediction, etc. China has a vast territory and complex geological conditions, and the natural geological environment that promotes geological disasters is also complex [1]. At present, the total number of major stations in various disaster monitoring systems in China has reached more than 43,000, and their geographical distribution is relatively scattered [2]. The early earthquake prediction research needs to describe dynamic natural factors at each station level, which makes the prediction of geographical location. Accuracy and efficiency cannot be guaranteed [3]. Based on GIS, the dynamic information of existing stations can be centrally managed [4], and the data analysis ability of dynamic information has been greatly improved, providing powerful conditions for the development of earthquake monitoring work.

Collecting seismic data to carry out its related identification work, industry-related personnel have carried out research on various automatic earthquake identification algorithms based on this field [5, 6], ratio represents the changes of signal amplitude, frequency, etc., this method will miss some signals with low bath ratio [7]; based on the Akaike information criterion method, the minimum point of the waveform curve is sought as the arrival time point of the earthquake relative, this method strongly depends on the signal-noise ratio and monitoring interval [8]; waveform correlation analysis method can monitor geology from a single area with the same focal mechanism [9], that is, it is more effective for repeated earthquake detection, and the detection accuracy depends on the number of samples used, but the larger the number of samples, the faster the amount of computation. The disadvantages of traditional seismic facies identification are heavy workload, long interpretation time, strong subjectivity, and low efficiency. Therefore, some seismologists pay more attention to automatic seismic interpretation. The use of intelligent geophysical technology can effectively improve the traditional seismic data processing, interpretation efficiency and result quality. The main technologies include big data, machine learning, and deep learning. Machine learning is used in geophysical data processing, rock physical property analysis, wellbore, reservoir, and oil and gas development data, but most of the current research and analysis are basically applied to seismic data processing. With the improvement of computer hardware and the breakthrough of big data computing performance, the deep learning technology represented by deep convolution neural networks has attracted the research interest of seismic interpretation workers in the field of seismic type identification.

A neural network algorithm is a class of algorithms implemented by simulating the way the human brain learns [10, 11]. “Neurons” represent nonlinear and correlated variables, which form a whole with a network structure, and construct a set of input features (such as seismic waveforms). Complex nonlinear relationship between expected output values (type of seismic phase), and based on the obtained relationship to predict the features of the new input, similar to pattern matching [12], the neural network extracts sample data from different seismic waveforms to generate Generalization performance of the model. This study uses GIS to collect 14,000 and 8,800 earthquake aftershock events manually selected from 30 stations in Sichuan and adjacent areas during July and August after the Wenchuan earthquake as the data training set and event test set, respectively. Analysis, compare the CNN model with other traditional models and then analyze the performance of missed aftershock events based on the model.

## 2. Acquisition of Seismic Waveform Data and Data Scene Fitting Test

Using the secondary development function of GIS and the Hilbert-Huang transform (HHT), the seismic waveform signal processing by this method is generally divided into two steps. First, EMD [13, 14] is used to obtain the multiple intrinsic mode function (IMF) [15]; the time series variable is transformed by Hilbert, and the frequency variable is calculated by instantaneous frequency to obtain the corresponding spectral curve. Considering that the instantaneous frequency only has an analytical value for single-component signals, in the acquisition of seismic data, the physical signal contains many other interference signals, which cannot be directly used for instantaneous frequency calculation, and these physical signals need to be approximated, as shown in Figure 1.

The signal is decomposed into multiple single-component signals by EMD, and can also be decomposed into the sum of mixed signals containing physical information components. From the perspective of execution, the upper and lower values of the physical signal to be measured need to be obtained first; The value is interpolated through multiple fittings, so that the upper limit of the signal is functionalized (*X*_max(*t*)_) and the lower limit is functionalized (*X*_min(*t*)_). Average as many points as possible to get the function *X*_mid(*t*)_.

Based on this method for seismic physical waveform signal acquisition, there will be obvious errors due to the influence of noise in the mechanical measurement. When calculating the point average value of each function, errors will also occur in the model itself. Because of the breakpoint phenomenon, using EMD to decompose itself also Various computational flaws will arise. After analyzing the signal intercepted by GIS, it can be seen that the Hilbert–Huang transformation can be used to process nonlinear and non-stationary signals. After analysis, the maximum amplitude corresponds to the period (*T*_max_), the cepstral mean value (Midcave), and the autocorrelation function. The maximum value (Maxcov) can represent the information of the waveform. The seismic scene has certain characteristics. Based on the intercepted data, the effectiveness of intercepting seismic vibration bands can be verified. GIS is used to screen some seismic data, and a seismic model is constructed in the shallow layer of the Loess Plateau. The sample interval of the model is 2 ms, and the main frequency of the source wavelet and the number of channels are 50 Hz and 400, respectively.  Table 1 sets other geological parameters of the model.

The effective geological waveform is used as a template to map to the surface wave test. The shallow bottom signal is concentrated in the *x* and *z* components. In addition to the surface wave information, there are also multiple wave information. After data simulation, a large number of *x* and *z* components are distributed in the part above the near-migration. Surface wave data, that is, the signal strength in this area is obvious.

## 3. CNN Algorithm Performance and Its Seismic Continuous Waveform Detection

### 3.1. CNN Network Structure

In the seismic waveform-noise classification analysis, the CNN structure is introduced [16], which has been cited in many studies and improved based on this structure. The purpose of CNN is to extract the features of things with a certain model, and then classify, recognize, predict or make decisions according to the features. The most important step is feature extraction, that is, how to extract features that can distinguish things to the greatest extent, and how to realize this great model requires iterative training for CNN. The model has translation invariance, that is, slightly changing the orientation or position of the same object may not activate the neurons that recognize the object; The existence of the pooling layer will lead to the loss of much valuable information, and will also ignore the association between the whole and parts. In this study, a CNN structure with the best performance in the problem of handwritten digit classification is used, as shown in Figure 2:

In the chosen CNN architecture, the convolutional layer can be used to achieve feature extraction [17, 18], and the pooling layer reduces the number of sample features to be tested through dimensionality reduction [19]. The two-dimensional convolution structure is common in the classification of handwritten digital images, and the seismic waveform data is not suitable for this method. The internal convolution kernel and channel are set to [3, 32], 4000 × 3 is used as the training input, and the three-component waveform is used as the waveform interval. After layer-by-layer peeling, it is converted into a one-dimensional feature of 20 × 32. After these features go through the fully connected layer, the ReLU activation function is used to calculate the probability of each waveform category to be classified, and it is compared with the preset classification threshold. If it is lower than the threshold, it will be marked as −1, that is, noise. If it is higher than the threshold, is marked with a value greater than 0, indicating an earthquake.

### 3.2. Preprocessing of Seismic Waveform Data Collected by GIS

In 2008, a magnitude 8.0 earthquake occurred in a county-level area called Wenchuan in Sichuan Province, China. The loss of people and property caused by the earthquake was huge. At the same time, aftershocks were frequent and the aftershocks were distributed in a wide area, with a magnitude of 0.2∼3.6. There are many large-scale aftershocks. At the same time, many researchers have carried out a large number of geological inspections in the area, recorded the aftershocks and obtained a large amount of data, so as to provide the original data for model training and waveform classification of this study.

The use of CNN for data analysis requires a large amount of data. Fewer samples will affect the recognition ability of the training model, and at the same time, it is prone to overfitting. An ideal data set needs a large amount of sample data for each category, so as to cover the complex features of seismic waveforms. The earthquake occurred at 30 stations in Sichuan and its adjacent areas, and the time was set between July and August. The data training set was 14,000 earthquake aftershock events that were manually selected, and 8,800 events were used for model testing. All event waveforms are taken from 8s before the arrival of P to 10s after the arrival of S. In terms of noise, random screening is adopted after excluding event waveforms. All data samples are waveform data within 30 s, and manual event labeling is reduced [20], Errors generated by noise are randomly screened [21], and easily found labeling errors are manually corrected. To increase the data, the enhancement method is an ideal method, and the one-dimensional three-channel image is used as the data format of the seismic waveform, which is realized by the methods of phase shifting, pixel blurring and filtering.

### 3.3. Algorithm Performance of CNN

Figure 3 shows the training and loss function curves of the preprocessed GIS seismic waveform data. It can be seen that the processed data set can converge faster.

In all algorithms, in order to minimize the cross-entropy loss function, L2 regularization and stochastic gradient descent are performed on the physical data of the training waveform, and the ADAM algorithm is used for optimization, thereby improving the calculation speed of data features. In the model training process of deep learning, the data involved in the training is iterated in one cycle called epoch [22]. Using Tensorflow to train 10 epochs on a 1080ti GPU only takes 15mn, and the average calculation accuracy during training exceeds 95%. In the recognition calculation of 8800 samples in the test set, it is found that the test samples can be recognized in less than 20s, and the training accuracy reaches 94.7%, as shown in Figure 3.

### 3.4. Comparison of Continuous Physical Waveform Detection based on GIS-CNN

In the experiment, the CNN model with the highest accuracy in the training set and test set is used for the detection of continuous physical waveforms, and the model is used for waveform recognition and comparison with the classical fbpicker algorithm [23] and STA/LTA algorithm [24]. The imported data comes from the continuous waveforms from August 1, 2008, to September 1, 2008, obtained by the MXI station of Sichuan Network. In order to verify that the model can improve the missed detection rate of aftershocks, the operation of manually selecting event waveforms is performed in the corresponding time period and 1805 events were selected for reference.

The precision *T* and recall rate *R* are selected to represent the recognition performance of different algorithms [25], and two subscripts are set for the corresponding indicators, namely noise and event:

(1) Te=MsMs+Ls,Re=MsMs+Ln.

Among them, the subscript *e* represents the event, the subscript *n* represents the noise, *Ms* represents the true case, that is, the event recognized by the algorithm is real, otherwise, there is a false case *Ls*, Mn represents the reverse case, that is, the waveform noise recognized by the algorithm is real On the contrary, there is a false reverse case, that is, *Ln*. The lower the false detection rate, the higher the recognition accuracy of the algorithm, and the lower the missed detection rate, the higher the corresponding recall rate. When evaluating the efficiency of the algorithm, the above two indicators need to be considered at the same time in order to verify whether the model has application value.

The precision and recall rate of different identification methods are listed in Table 2. Among them, CNN identified 3767 aftershock event waveforms, of which 1805 events were consistent with the number of reference samples. Compared with the CNN method, the traditional identification algorithm had better precision and recall rate. Neither is as good as the former.

It should be noted that the manual aftershock waveform samples selected for reference have undergone seismic positioning and correlation processing, so they have high accuracy. However, due to the limitations and subjectivity of human identification, the data lacks integrity, such as isolated events or signal-to-noise. Aftershock events smaller than the soles of the feet are easily missed. Relevant studies have confirmed that the CNN structure can identify aftershocks and even small microseisms in the process of earthquake waveform classification. Based on this, in the calculation process of *Te*, there are many types of events that need to be considered, not just defined as *Ls*, so it cannot be very good. It reflects the classification effect of the CNN algorithm.

In Figure 4, the continuous physical waveform of the MXI station on August 23, 2008, was identified as the data source. There were 50 manually selected events on that day, but through further observation, it was found that there were about 370 small aftershocks with smaller amplitudes on that day (Figure 4(a)). These small aftershocks can be better identified by CNN (Figure 4(b)), and when these missed aftershocks are included, the precision and recall of the algorithm reach 73.7% and 62.8%, respectively. After being processed by the CNN model, the misclassified waveform data can be substituted into the training as part of the metadata, so as to better distinguish different seismic waveforms.

## 4. Conclusion

The Hilbert-Huang transform (HHT) has advantages in dealing with nonlinear and non-stationary problems. In this study, this transformation is first performed on the GIS intercepted data, so that the collected data is not restricted by linearity and stationarity, and can be used for nonlinear Analysis of non-stationary physical signals. HHT is self-adaptive but does not have the ability to distinguish signals in the time domain. The conversion can generate corresponding databases according to the requirements of the problem, that is, generate the required IMFs. HHT is suitable for mutation signals and is not restricted by the Heisenberg uncertainty principle. The instantaneous frequency is obtained by derivation, and the phase function is obtained by using the Hilbert transform. Further derivation is used to calculate the instantaneous frequency. The result of this index only acts on the local fragment of the signal. Using GIS to intercept data from seismic raw physical waveform data is only the first step. At the same time as data preprocessing, the CNN method is introduced. Compared with the traditional identification method of single or multiple feature functions, the use of CNN can greatly improve the classification accuracy to be tested. At the same time, the model has a relatively stable output effect. Different from the waveform similarity method, the CNN obtains the feature of the drawn line from the training data set and is not based on the waveform amplitude, so it has better model coverage [26].

## Figures and Tables

**Figure 1:** GIS-based seismic data acquisition process.

**Figure 2:** The structure of the convolutional neural network used.

**Figure 3:** The training process before and after data preprocessing, (a) training curve, (b) cross-entropy loss function curve.

**Figure 4:** Example of CNN continuous physical waveform detection with manual samples. (a) Black balls indicate manually picked events and red balls indicate manually missed small aftershock events. (b) Event fragments identified by the CNN algorithm.

**Table 1:** Some parameters of the simulated geological model.

	Layer thickness (m)	Poisson's ratio	Shear wave velocity *Vs* (m/s)	Longitudinal wave velocity *Vp* (m/s)	Density
1	3	0.35	180	380	1.6
2	5	0.40	260	760	1.68
3	10	0.45	265	880	1.73
4	20	0.40	400	1010	1.8

**Table 2:** Comparison of CNN and traditional recognition (fbpicker, STA/LTA) algorithms.

Method	*Te*	*Re*	*Ms*	*Ls*	*Ln*
CNN	48.1% (1805/3757)	95.4% (1805/1891)	1805	1952	86

Fbpicker	29.2% (1589/5446)	85.3% (1589/1863)	1589	3857	274

STA/LTA	36% (1666/4633)	87.6% (1666/1902)	1666	2967	236

## Data Availability

The dataset used in this paper is available from the corresponding author upon request.
